This article has been retracted.

# Effect of Shenqi Fuzheng Injection on Leukopenia and T-cell Subsets in Patients with Non-small Cell Lung Cancer Undergoing Radiotherapy

**DOI:** 10.1155/2022/2832739

**Published:** 2022-08-05

**Authors:** Chengde Wu, Ying Liang, Fangyong Fu

**Affiliations:** Department of Thoracic Surgery, Central South University Xiangya School of Medicine Affiliated Haikou Hospital, Haikou 570208, China

## Abstract

**Purpose:**

The aim of this study is to evaluate the effect of Shenqi fuzheng injection on leukopenia and T-cell subsets in patients with non-small cell lung cancer (NSCLC) undergoing radiotherapy.

**Methods:**

A total of 124 patients with advanced NSCLC treated in the oncology department of our hospital from January 2017 to January 2019 were included and assigned at a ratio of 1 : 1 to receive conventional radiotherapy (control group, *n* = 62) or conventional radiotherapy plus Shenqi Fuzheng injection (study group, *n* = 62) via the random number table method.

**Results:**

The study group showed a significantly higher objective response rate (ORR) and a lower incidence of leukopenia versus the control group (*P* < 0.05). After the treatment, Shenqi Fuzheng injection resulted in significantly lower levels of carcinoembryonic antigen (CEA) and neuron-specific enolase (NSE) in the study group versus conventional treatment given to the control group. After the treatment, the control group showed significantly decreased ratios of CD3+ T cells, CD4+ T cells, and CD4+/CD8+, and an increased ratio of CD8+ T cells, and significant differences when compared with the study group. The T-cell subsets of the patients in the study group showed no significant changes than those between the treatment. The median OS was 20.0 months in the control group and 23.5 months in the study group. The differences between the two groups in terms of OS did not come up to the statistical standard.

**Conclusion:**

Shenqi Fuzheng injection for NSCLC patients undergoing radiotherapy elevates the number of white blood cells, regulates T-cell immune function, reduces tumor markers, and enhances clinical efficacy. Further clinical trials are, however, required prior to clinical promotion.

## 1. Introduction

Lung cancer is a common malignant tumor with a high prevalence and mortality, and its symptoms include cough, sputum, hemoptysis, and chest pain [1]. In 2020, the number of new cancer cases worldwide was 19,292,789, of which 4,568,754 (about 4.56 million) were new cases of cancer in China, accounting for 23.7% of the world's total. The increase in the incidence of lung cancer is closely related to environmental pollution, population aging, and unhealthy lifestyles [2]. Mortality from lung cancer is mainly attributed to distant metastasis despite surgical resection with curative intent. Moreover, due to the insidious symptoms at the early stage, lung cancer patients are mostly diagnosed at the advanced stage [3], where conservative treatments such as radiotherapy and chemotherapy are mainly adopted for disease control. However, chemoradiotherapy causes collateral damage to the adjacent normal tissues and results in reduced therapeutic effects [4]. Thus, there exists a need to explore effective treatment methods to prolong patient survival and enhance the quality of life. NSCLC is a common type of lung cancer, and chemotherapy based on cytotoxic drugs is a common treatment for patients with advanced lung cancer. However, chemotherapy seriously affects the immunity of the body and their quality of life and is prone to drug resistance.

According to traditional Chinese medicine (TCM), lung cancer is mainly caused by stagnation of qi and blood in the lung promoted by internal deficiency of positive qi and external invasion of evil toxins. In advanced cancer patients, the deficiency of positive qi and the prevailing evil toxins may lead to insufficient body resistance against the evil qi and further depletion of positive qi, resulting in disease aggravation [5, 6]. Therefore, maintenance of positive qi and a combination of tumor cell killing with immunity reinforcement is the key to treatment [7]. The application of traditional Chinese medicine in lung cancer has been widely reported, and the adjuvant therapy of traditional Chinese medicine plays the role in relieving postoperative adverse reactions and enhancing the immune function of the body. Studies have shown that the combination of Sun-Bai-Pi extract and cisplatin can produce a synergistic effect, improve the killing effect of chemotherapy drugs on lung cancer cells, and promote the rapid clearance of tumor cells. The effects of single traditional Chinese medicines such as tanshinone, cinnamaldehyde, and puerarin in inducing tumor cell apoptosis have also been confirmed [8]. Shenqi Fuzheng injection is a classic TCM preparation, mainly containing Astragali Radix and Codonopsis Radix, both of which are tonic medicines that benefit the spleen and lung meridians, nourish the middle Jiao, activate the body's positive qi, improve the patient's immunity, and alleviate the adverse consequences of radiotherapy [9]. Astragali Radix is the root of *Astragalus membranaceus* (Fisch.) Bunge and is sweet in taste with mild heat. It nourishes the spleen and lung meridians, improves the body's immune function, and regulates the balance of qi and blood in the internal organs of the body tonifying the qi, strengthening the spleen, enhancing the Yang, and reducing swelling [10, 11]. Relevant research proved that ginseng polysaccharide, which is rich in Codonopsis Radix, exhibits low toxicity and strong pharmacological activity with anticancer effects [12]. The present study was undertaken to evaluate the effect of Shenqi fuzheng injection on leukopenia and T-cell subsets in patients with non-small cell lung cancer (NSCLC) undergoing radiotherapy, so as to provide a reference for further research on the clinical indications of Shenqi Fuzheng injection and to reveal its pharmacological mechanism of action.

## 2. Materials and Methods

### 2.1. Participants

A total of 124 patients with advanced NSCLC treated in the oncology department of our hospital from January 2017 to January 2019 were included and assigned at a ratio of 1 :  1 to receive conventional radiotherapy (control group, *n* = 62) or conventional radiotherapy plus Shenqi Fuzheng injection (study group, *n* = 62) via the random number table method. The study was approved by the ethics committee of Central South University Xiangya School of Medicine Affiliated Haikou Hospital and followed the Declaration of Helsinki ethical guidelines for clinical trials [13]. Undersigned informed consent was obtained from the participants and their families for this study.

### 2.2. Inclusion and Exclusion Criteria

#### 2.2.1. Inclusion Criteria

Patients who were aged 18–80 years, who were pathologically diagnosed with non-small cell lung cancer with clinical stage IIIB-IV, without surgical indication, with at least one measurable lesion, with an expected survival of ≥3 months, with no previous radiation therapy and tolerance to chemotherapy were included.

#### 2.2.2. Exclusion Criteria

Patients with malignant neoplastic diseases at other sites, with active infectious disease or presence of acute inflammatory disease requiring systemic treatment, who were pregnant or lactating women, with childbirth plans during the study period, with communication difficulties that prevent timely follow-up, and with other diseases such as severe liver, kidney, and other organ dysfunction were excluded.

### 2.3. Treatment Methods

All patients received three-dimensional conformal radiotherapy with the Novalis Tx (NTX) linear accelerator. The target areas of radiotherapy included the primary foci, the ipsilateral lung hilum, and the involved lymphatic drainage area. Patients received radical prescription doses within 6∼7 weeks, totaling 60–70 Gy, 2 Gy/dose. The maximum dose for the spinal cord was within 45 Gy, the average dose for the esophagus was within 34 Gy, and the maximum dose for the brachial plexus was within 66 Gy. Patients in the study group received 250 mL of Shenqi Fuzheng injection (Lizhu Group Limin Pharmaceutical Factory, approval number: Z19990065) on day 1 of radiotherapy through intravenous infusion daily, with a course of 21 d for a total of 2 courses.

### 2.4. Outcome Measures

#### 2.4.1. Clinical Efficacy

At 4 weeks after radiotherapy, the Response Evaluation Criteria in Solid Tumors (RECIST) [14] was used to classify the outcome into complete remission (CR), partial remission (PR), stable disease (SD), and progressive disease (PD).

PR indicates the complete disappearance of lesions on imaging. CR indicates a reduction of >50% of the lesions on imaging without the appearance of new lesions. SD indicates a reduction of 25–50% of the lesions on imaging without the appearance of new lesions. PD indicates a reduction of less than 25% of the lesions on imaging or the appearance of new lesions. Objective Remission Rate (ORR) = PR + CR/total cases^*∗*^100%.

#### 2.4.2. Leukocyte Count

On day 7 after radiotherapy, patients underwent routine blood tests. According to the WHO myelosuppression criteria [15], leukopenia was classified into grades 0 to IV, with grade 0 for leukocytes ≥4.0 × 109/L, grade I for leukocytes (3.0–3.9) × 109/L, grade II for leukocytes (2.0–2.9) × 109/L, grade III for leukocytes (1.0–1.9) × 109/L, and grade IV for leukocytes ≤1.0 × 109/L.

#### 2.4.3. Tumor Markers

Fasting venous blood was collected from patients before and after treatment, and the levels of carcinoembryonic antigen (CEA) and neuron-specific enolase (NSE) were determined by electrochemiluminescence.

#### 2.4.4. Peripheral Blood T-cell Subsets

Fasting venous blood was collected from patients before and after treatment, respectively, and the ratios of circulating CD3+ T cells, CD4+ T cells, and CD8+ T cells were determined by flow cytometry, and the CD4+/CD8+ were calculated.

#### 2.4.5. Long-Term Therapeutic Effects

Patients were followed up for 3 years after surgery, starting from the 2nd month after discharge with a follow-up visit every 2 months. Adverse reactions and survival status during the follow-up period were recorded.

### 2.5. Statistical Analysis

SPSS 22.0 was used for data organization and statistical analyses, and *R* language was used to plot the graphics. The measurement data were tested for normality, and non-normal data were converted to normal data by using Box-Cox Transformation. The measurement data are expressed as mean ± standard deviation (*x̅* ± *s*) and analyzed using the *t*-test. Count data are expressed as rates (%) and analyzed using the chi-square test. Survival data were tested using the K–M test and survival curves were plotted. The difference was considered statistically significant with *α* = 0.05 as the limit of significance.

## 3. Results

### 3.1. Patient Characteristics

The patient characteristics between the two groups, such as gender, age, KPS score, pathological type, and TNM stage, were not statistically significant and were comparable (all *P* < 0.05). (Table 1).

### 3.2. Clinical Efficacy

In the control group, there were 16 cases of CR, 18 cases of PR, 24 cases of SD, and 4 cases of PD, with an ORR of 54.84% (34/62). In the study group, there were 24 cases of CR, 22 cases of PR, 14 cases of SD, and 2 cases of PD, with an ORR of 74.19% (46/62). The ORR of the study group was significantly higher than that of the control group (*χ*^2^ = 5.073, *P*=0.024). (Table 2).

### 3.3. Leukocyte Count

In the control group, there were 22 cases of grade 0, 28 cases of grade I, 11 cases of grade II, 1 case of grade III, and 0 cases of grade IV, and the incidence of leukopenia was 64.52% (40/62). In the study group, there were 38 cases of grade 0, 18 cases of grade I, 6 cases of grade II, 0 cases of grade III, and 0 cases of grade IV, and the incidence of leukopenia was 38.71% (24/62). Patients in the study group showed a significantly lower incidence of leukopenia versus those in the control group (*χ*2 = 8.267, *P*=0.004). (Table 3).

### 3.4. Tumor Marker Levels

Before the treatment, there was no significant difference in the levels of CEA and NSE between the two groups (*P* > 0.05). After the treatment, patients receiving Shenqi Fuzheng injection in the study group were associated with significantly lower levels of CES and NSE versus those in the control group (*P* < 0.05). (Table 4).

### 3.5. T-cell Subsets

Before the treatment, the differences in the ratio of CD3+ T cells, the ratio of CD4+ T cells, the ratio of CD8+ T cells, and the CD4+/CD8+ ratio between the two groups were not statistically significant (all *P* > 0.05). After the treatment, the control group showed significantly decreased ratios of CD3+ T cells, CD4+ T cells, and CD4+/CD8+, and an increased ratio of CD8+ T cells, and significant differences when compared with the study group (all *P* < 0.05). The T-cell subsets of the patients in the study group showed no significant changes than those between the treatment (*P* > 0.05). (Table 5).

### 3.6. Overall Survival

The median OS was 20.0 months (95% CI: 18, 24) in the control group and 23.5 months (95% CI: 19.0, 30.0) in the study group. The differences between the two groups in terms of OS did not come up to the statistical standard (Table 6 and Figure 1).

## 4. Discussion

Lung cancer is a malignant tumor with high prevalence, and the long-term survival of patients remains poor despite the continuous improvement of treatment protocols [16]. In recent years, the role of TCM in adjuvant therapy against cancer has received increasing recognition [17].

Leukopenia is a common complication of chemoradiotherapy and may lead to serious complications such as secondary infections [18]. The results of the present study demonstrated that Shenqi Fuzheng injection could significantly alleviate serum leukopenia in lung cancer patients under radiotherapy. Oncogenesis impairs the function of the hematopoietic system, and myelosuppression occurs during chemoradiotherapy, which compromises the therapeutic effect and even threatens the life of the patient [19]. It has been reported that Shenqi Fuzheng injection plus granulocyte colony-stimulating factor was effective in managing leukopenia in acute leukemia by mitigating oxidative stress and improving survival quality [20]. In addition, a relevant study confirmed that Shenqi Fuzheng injection could significantly reverse patients' qi deficiency, enhance immune function, improve treatment effect and quality of life, and prolong their survival time [21]. CEA and NSE are common markers of NSCLS and play an important role in tumor diagnosis, clinical treatment, and prognostic assessment, and an increase in their expression levels suggests a poor prognosis [22]. In the present study, patients in the study group showed significantly lower levels of CEA and NSE, suggesting that Shenqi Fuzheng injection improved the prognosis of patients, which may be attributed to the fact that *Astragali radix* and *Codonopsis radix* enhanced the sensitivity of tumor cells to radiotherapy, which indirectly boosted the effectiveness of radiotherapy. Using proteomics and phosphorylation modification omics and other technologies, the tumor suppressor effect of some traditional Chinese medicine components was revealed. The researchers conducted quantitative proteomics and phosphorylation modification group of non-small cell lung cancer A549 cell line treated with ginsenoside extract. Through scientific analysis, it was found that Ras protein plays a regulatory role in multiple functional pathways, indicating that it is likely to be the target protein of a certain component of ginsenosides [23]. In addition, it was verified that bruceine *D* (Bruceine D), by targeting ICAT, blocked the interaction between ICAT and *β*-catenin, promoted the degradation of *β*-catenin in liver cancer cells, and then down-regulated HIF-1*α* and its downstream glucose metabolism expression of related genes in hypoxic liver cancer cells, and ultimately inhibited the energy metabolism of liver cancer cells and the growth of tumors in vivo. However, the composition of traditional Chinese medicine prescriptions is complex, and there are few related proteomic studies [24].

Chemotherapy and radiotherapy can render tumor cells visible to the immune system but also lower the number of immune cells and impair the immunity of the body. T lymphocyte subsets, including CD4+ T lymphocytes and CD8+ T lymphocytes, play a dominant role in the cellular immune response. CD4+ T lymphocytes are helper T cells with antitumor effects and CD8+ T lymphocytes are cytotoxic T cells whose increase facilitates continued tumor growth and promotes tumor cell proliferation, both of which collectively maintain immune function. CD4+/CD8+ downregulation is associated with reduced immunity [25]. It has been found that radiotherapy-induced reduction in T lymphocytes, especially CD4+ T cells, is associated with a poor prognosis of cancer. Clinical studies have shown that Shenqi Fuzheng injection stimulates bone marrow hematopoiesis, enhances body immunity, potentiates efficiency, and reduces toxicity in anticancer treatment [26]. In the present study, the CD3+ T cells, CD4+ T cells, CD5+ T cells, and CD4+/CD8+ ratio in the study group were significantly higher than those in the control group, indicating that Shenqi Fuzheng injection enhanced the immune function of lung cancer patients under radiotherapy. However, the specific mechanism is not analyzed and discussed in this paper. Most of the references in this article are clinical studies, lacking evidence support from basic studies.

## 5. Conclusion

Shenqi Fuzheng injection for NSCLC patients undergoing radiotherapy elevates the number of white blood cells, regulates T-cell immune function, reduces tumor markers, and enhances clinical efficacy. Further clinical trials are, however, required prior to clinical promotion.

## Figures and Tables

**Figure 1:** Overall survival.

**Table 1:** Patient characteristics.

	Control group (*n* = 62)	Study group (*n* = 62)	*t/χ * ^2^	*P* value
*Gender*			0.308	0.579
Male	40	37		
Female	22	25		
*Age*	67.15 ± 13.21	65.18 ± 15.43	0.764	0.447
*KPS score*			0.175	0.676
≥80 points	34	36		
<80 points	18	16		
*Pathological type*			0.831	0.660
Squamous cell carcinoma	22	20		
Adenocarcinoma	30	28		
Others	10	14		
*TNM stage*			0.314	0.575
III	21	24		
IV	41	38		

**Table 2:** Clinical efficacy (*n*, %).

	*n*	CR	PR	SD	PD	ORR
Control group	62	16 (25.81)	18 (29.03)	24 (38.71)	4 (6.45)	34 (54.84)
Study group	62	24 (38.71)	22 (35.48)	14 (22.58)	2 (3.23)	46 (74.19)
*χ * ^2^						5.073
*P* value						0.024

**Table 3:** Leukocyte count (*n*, %).

	*n*	Grade 0	Grade I	Grade II	Grade III	Grade IV	Total incidence
Control group	62	22	28	11	1	0	40 (64.52)
Study group	62	38	18	6	0	0	24 (38.71)
*χ * ^2^							8.267
*P* value							0.004

**Table 4:** Tumor marker levels ($\bar{x}$ ± *s*, *n*g/mL).

	*n*	CEA		NSE	
		Before	After	Before	After
Control group	62	51.93 ± 7.21	46.44 ± 6.36	27.14 ± 4.55	23.45 ± 4.16
Study group	62	50.81 ± 9.13	41.15 ± 7.43	26.16 ± 5.02	21.03 ± 4.08
*t* value		0.758	4.259	1.139	3.270
*P* value		0.450	<0.001	0.257	0.001

**Table 5:** T-cell subsets ($\bar{x}$ ± *s*).

	*n*	CD3+T (%)		CD4+T (%)		CD8+T (%)		CD4+/CD8+	
		Before	After	Before	After	Before	After	Before	After
Control group	62	56.11 ± 10.14	50.15 ± 8.24^#^	33.15 ± 7.24	28.45 ± 6.31^#^	24.15 ± 4.31	27.49 ± 5.40^#^	1.51 ± 0.35	1.26 ± 0.28^#^
Study group	62	55.72 ± 11.53	54.48 ± 9.25	32.81 ± 7.37	31.83 ± 7.17	25.33 ± 5.02	24.15 ± 4.92	1.53 ± 0.31	1.48 ± 0.29
*t* value		0.200	2.752	0.259	2.786	1.404	3.600	0.337	4.297
*P* value		0.842	0.007	0.780	0.006	0.162	<0.001	0.737	<0.001

^#^indicates *P* < 0.05 when compared to the same group before treatment.

**Table 6:** Overall survival.

	*n*	Median survival	95%CI
Control group	62	20.0	18.0 ∼ 24.0
Study group	62	23.5	19.0 ∼ 30.0
HR		1.396	0.938 ∼ 2.077
*P* value		0.089	

## Data Availability

All data generated or analyzed during this study are included in this published article.

## References

[1] Nasim F., Sabath B. F., Eapen G. A. (2019). Lung cancer. *Medical Clinics of North America*.

[2] Hoy H., Lynch T., Beck M. (2019). Surgical treatment of lung cancer. *Critical Care Nursing Clinics of North America*.

[3] Shintani R., Sekine A., Murohashi K. (2022). Successful treatment of chylothorax and chylopericardium by radiotherapy in lung cancer. *Internal Medicine*.

[4] Deng L., Harðardottír H., Song H. (2019). Mortality of lung cancer as a second primary malignancy: a population-based cohort study. *Cancer Medicine*.

[5] Su X. L., Wang J. W., Che H. (2020). Clinical application and mechanism of traditional Chinese medicine in treatment of lung cancer. *Chinese Medical Journal*.

[6] Wang K., Chen Q., Shao Y. (2021). Anticancer activities of TCM and their active components against tumor metastasis. *Biomedicine & Pharmacotherapy*.

[7] Li Z., Feiyue Z., Gaofeng L. (2021). Traditional Chinese medicine and lung cancer-From theory to practice. *Biomedicine & Pharmacotherapy*.

[8] Qi F., Zhao L., Zhou A. (2015). The advantages of using traditional Chinese medicine as an adjunctive therapy in the whole course of cancer treatment instead of only terminal stage of cancer. *BioScience Trends*.

[9] Dong J., Su S. Y., Wang M. Y., Zhan Z. (2010). Shenqi fuzheng, an injection concocted from Chinese medicinal herbs, combined with platinum-based chemotherapy for advanced non-small cell lung cancer: a systematic review. *Journal of Experimental & Clinical Cancer Research*.

[10] Chen Z., Liu L., Gao C. (2020). Astragali Radix (Huangqi): a promising edible immunomodulatory herbal medicine. *Journal of Ethnopharmacology*.

[11] Shahzad M., Shabbir A., Wojcikowski K., Wohlmuth H., C Gobe G. (2016). The antioxidant effects of Radix Astragali (Astragalus membranaceus and related species) in protecting tissues from injury and disease. *Current Drug Targets*.

[12] Luan F., Ji Y., Peng L. (2021). Extraction, purification, structural characteristics and biological properties of the polysaccharides from Codonopsis pilosula: a review. *Carbohydrate Polymers*.

[13] Malik A. Y., Foster C. (2016). The revised Declaration of Helsinki: cosmetic or real change?. *Journal of the Royal Society of Medicine*.

[14] Schwartz L. H., Seymour L., Litière S. (2016). Recist 1.1-standardisation and disease-specific adaptations: perspectives from the RECIST working group. *European Journal of Cancer*.

[15] He M., Wang N., Zheng W. (2021). Ameliorative effects of ginsenosides on myelosuppression induced by chemotherapy or radiotherapy. *Journal of Ethnopharmacology*.

[16] Cao W., Chen H. D., Yu Y. W., Li N., Chen W. Q. (2021). Changing profiles of cancer burden worldwide and in China: a secondary analysis of the global cancer statistics 2020. *Chinese Medical Journal*.

[17] Chen D. M., Mao K. Y., Yang L., Jiang H. B. (2014). Status of anti-lung cancer drug patents applications in China from 2003 to 2012. *Recent Patents on Anti-cancer Drug Discovery*.

[18] Zhou J. G., Tian X., Cheng L. (2015). The risk of neutropenia and leukopenia in advanced non-small cell lung cancer patients treated with erlotinib: a prisma-compliant systematic review and meta-analysis. *Medicine (Baltimore)*.

[19] Joseph N., Choudhury A. (2021). Dosimetric predictors of radiotherapy-induced lymphocytopenia in lung cancer. *Journal of Thoracic Oncology*.

[20] Meng F. X., Yang X., Li M. L. (2022). Shenqi fuzheng injection combined with chemotherapy for acute leukemia: a meta-analysis. *Chinese Journal of Integrative Medicine*.

[21] Du J., Cheng B. C. Y., Fu X. Q. (2016). In vitro assays suggest Shenqi Fuzheng Injection has the potential to alter melanoma immune microenvironment. *Journal of Ethnopharmacology*.

[22] Li Q., Sang S. (2020). Diagnostic value and clinical significance of combined detection of serum markers CYFRA21-1, SCC Ag, NSE, CEA and ProGRP in non-small cell lung carcinoma. *Clinical Laboratory*.

[23] Wang Z., Kim U., Jiao Y. (2019). Quantitative proteomics combined with affinity MS revealed the molecular mechanism of ginsenoside antitumor effects. *Journal of Proteome Research*.

[24] Huang R., Zhang L., Jin J. (2021 Nov). Bruceine D inhibits HIF-1*α*-mediated glucose metabolism in hepatocellular carcinoma by blocking ICAT/*β*-catenin interaction. *Acta Pharmaceutica Sinica B*.

[25] Chraa D., Naim A., Olive D., Badou A. (2019). T lymphocyte subsets in cancer immunity: friends or foes. *Journal of Leukocyte Biology*.

[26] Yang Y., Ting W., Xiao L. (2017). Immunoregulation of Shenqi fuzheng injection combined with chemotherapy in cancer patients: a systematic review and meta-analysis. *Evidence-based Complementary and Alternative Medicine*.

